The article "Efficacy of Mesotympanum Injection and Posterior Auricular Injection in Sudden Hearing Loss of Diabetes Patients" was retracted in 2024. Reasons: signs of a paper mill; compromised peer review; unreliable results or conclusions.

# Efficacy of Mesotympanum Injection and Posterior Auricular Injection in Sudden Hearing Loss of Diabetes Patients

**DOI:** 10.1155/2022/8494868

**Published:** 2022-07-19

**Authors:** Qiang Liu, HuiFang Wang, JiHuan Xing

**Affiliations:** E.N.T Department, Beichen Hospital, Tianjin, 300400 Tianjin, China

## Abstract

The efficacy of tympanum injection and posterior auricular injection in diabetes with sudden hearing loss (SHL) was analyzed. A mobile terminal-based portable pure tone audiometry system and its processing method were established. Based on mobile terminals, a portable pure tone audiometry system including an Android system, pure sound signal generation, pure tone hearing threshold, and client module was established. A masking model and self-adaptive algorithm were used to detect and reduce noise. Besides, the performance of the portable pure tone audiometry system was detected. A total of 46 diabetes patients with SHL diagnosed at the otolaryngology department in BeiChen Hospital between August 2019 and November 2021 were selected as the research objects and randomly divided into the retroauricular group (posterior auricular injection) and the tympanic group (tympanum injection). Each group included 23 cases. All patients received pure tone audiometry (PTA) before and after the treatment. The changes in fasting blood glucose (FPG), 2h postprandial blood glucose (2hPG), and glycosylated hemoglobin (HbA1c) of the patients were monitored before and after the treatment. Besides, tinnitus loudness visual analog scale (VAS), pain VAS, efficacy, and the incidence of adverse reactions of the patients in two groups were compared. The results indicated that the hear threshold error detected by the medical audiometer and a portable pure tone audiometry system was within 2dB. Before the optimization, there was an error of about 10dB between the hear thresholds detected by the self-adaptive algorithm and a medical audiometer. After the treatment, the hear threshold and average PTA of the patients in the retroauricular and the tympanic groups under different frequencies were both reduced compared with those before the treatment (*P* < 0.05). The tinnitus VAS score in the retroauricular group was decreased more notably than that in tympanic group (*P* < 0.01), and the pain VAS score was much lower than that in the tympanic group (*P* < 0.001). The comparison of FPG, 2hPG, HbA1c, the proportions of cured, significantly effective, effective, ineffective patients, and the total effective rate in the patients in the retroauricular and the tympanic groups before and after the treatment all showed no statistical differences (*P* > 0.05). The incidence of adverse reactions in tympanic group after the treatment was dramatically higher than that in retroauricular group (*P* < 0.001). The above results demonstrated that posterior auricular injection showed potential application values in the treatment of SHL with diabetes and established a portable pure tone audiometry system as well as its noise processing method.

## 1. Introduction

Sudden hearing loss (SHL) is a common otolaryngological acute symptom. SHL patients usually suffer from unexplained sensorineural hearing loss within minutes, hours, or 3 days. Hearing loss reaches over 30 dB at least two connected frequencies. Patients often suffer from tinnitus, vertigo, ear stuffy feeling, and other clinical symptoms [1]. According to the statistics, the annual incidence of SHL is as high as 160 per 100,000 [2]. The incidence of SHL among the population aged around 50 is high [3]. In recent years, SHL incidence shows an obvious ascending trend with the acceleration of people' life pace in recent years [4]. SHL causes a serious impact on people's quality of life and permanent hearing loss if patients are untreated timely. Some patients may suffer from persistent tinnitus and other sequelae [5]. At present, the pathogenesis of SHL is unknown. In clinical practice, glucocorticoid, antioxidant, anticoagulant drug, and neurotrophic drug are often utilized to treat SHL [6]. Diabetes is a common metabolic disease characterized by chronic hyperglycemia. Its complications may involve in each organ system. The current research results reveal that hyperglycemia, insulin resistance, lipid metabolism, and the changes in the expressions of cell factors and hormone cause impaired blood supply to the inner ear among diabetes patients. At the early stage of diabetes, minor damage to peripheral organs and dysfunction of the auditory center and peripheral nervous system may occur [7]. In some studies, it is pointed out that 16% of SHL patients suffer from combined diabetes [8]. The treatment of SHL patients with diabetes by glucocorticoid causes an increase in glyconeogenesis, the reduction in peripheral glucose utilization, and the aggravation of diabetes [9]. As a common drug for the clinical treatment of SHL, dexamethasone can be administered intravenously, in the tympanum, or in the posterior auricular tympanum [10]. Posterior auricular tympanum injection is a treatment scheme stated late. At present, there are few comparative studies on the efficacy of tympanum injection and posterior auricular tympanum injection in SHL with diabetes.

A pure tone audiometry (PTA) is a method of measuring absolute auditory threshold under specified conditions and one of the main clinical methods of determining auditory sensitivity [11]. The method shows significant values in the diagnosis of ear diseases, the evaluation of drug therapeutic effect, and the selection of rehabilitation measures. The existing commonly used clinical PTA methods include air conduction auditory threshold test, bone conduction auditory threshold test, and sound field audiometry method [12]. The adoption of these methods has high requirements on the test environment, test devices, and test personnel. With the continuous development of network communication and Internet technology in recent years, a portable intelligent device is gradually applied in a medical diagnostic system [13]. A portable PTA system can overcome the shortcomings of traditional PTA with simple operation and timely detection of ear hearing damage. Some researchers introduce wireless communication technology into remote hearing assessment system. Nonetheless, a portable PTA system is susceptible to environmental noise [14] and needs to be further optimized.

To sum up, there are few comparative studies on the efficacy of tympanum injection and posterior auricular tympanum injection in SHL with diabetes. A portable PTA system is susceptible to environmental noise and needs to be further optimized. Hence, a portable PTA system was established preliminarily based on mobile terminals. Besides, its noise processing method was discussed, and the efficacy of the tympanum injection and the posterior auricular tympanum injection in SHL with diabetes was compared to provide a new idea and reference basis for the diagnosis and treatment of SHL.

## 2. Materials and Methods

In the sections, we will discuss MTPPSD, methods of processing portable PTA system noise, research objects and grouping, different therapeutic methods for diabetes patients with SHL, judgment methods of efficacy and observation indexes, and statistical methods.

### 2.1. Mobile Terminal-Based Portable PTA System Design

Based on system functional requirement analysis, a mobile terminal-based portable PTA system mainly includes software and hardware parts. Software parts include an Android system, pure tone signal generation module, pure tone auditory threshold module, and client results display module. An Android system mainly involves Android operating system programming. According to frequency information, the pure tone signal survival module can generate a corresponding pure signal. Client results display module can show the audiogram and frequency resolution diagram of the subjects. Hardware parts mainly include sound card, graphics card, central processing unit (CPU), earphone, and hardware resources of mobile devices.  Figure 1 displays the overall framework of a mobile terminal-based portable PTA system below.

In the application of a mobile terminal-based portable PTA system, the distance and noise of different devices have different influences on the system. Hence, the influences of distance and noise on the system need to be analyzed before the application of the established a portable PTA system. Self-adaptive algorithm is used to detect and reduce the remaining noise. Besides, masking model is set up to remove noise interference to obtain the test noise after the denoising. After that, it is compared with relevant hospital medical devices. The test noise is calibrated to obtain relevant parameters. Next, the subjects' speech is tested to acquire the test tone.  Figure 2 shows the application process of a portable PTA system below.

### 2.2. Methods of Processing a Portable PTA System Noise

The intensity of the sound produced by sound source is correlated with noise [15]. Therefore, the influence of test distance on the monitoring results of portable PTA system needs to be analyzed before noise processing to determine the optimal test distance. The loud speaker of Android cellphone in the proposed portable PTA system is used as the main sound source with the size of 0.03 m × 0.01 m. It is assumed that the length of a surface sound source is *l* and its width is *w*. Besides, propagation distance is *d*. As a result, the attenuation of the sound source with distance meets the following conditions, as shown in the following equations.

(1) $$\begin{array}{c} d<\frac{w}{\pi },\;\text{SIA}\approx 0,\\ \frac{w}{\pi }<d<\frac{l}{\pi },\;\text{SIA}\approx 3\text{dB},\\ d>\frac{l}{\pi },\;\text{SIA}»6\text{dB}. \end{array}$$

In the above equations, SIA refers to sound intensity level attenuation. SIA ≈ 0 indicates that there is almost no attenuation of the intensity of the sound propagated. SIA ≈ 3 dB and SIA ≈ 6 dB mean that the attenuation values of sound intensity levels are about 3 dB and 6 dB, respectively, as propagation distance doubles.

The receiver of the sound source is human ears. The test distance refers to the distance from the loud speaker of Android cellphone to the center of two ears. The test reveals that human body can touch the device when the test distance ranges between 0.2 m and 0.6 m. As a result, the test distance is expressed by the following equation below.

(2) $$\begin{array}{c} 0.2\leq d\leq 0.6. \end{array}$$

The loud speaker of Android cellphone is viewed as the sound source, and the signal intensity monitored by human ears is expressed by the following equation below.

(3) $$\begin{array}{c} D\left(s\right)=D\left(s_{0}\right)-20\mathrm{lg}\left(\frac{s}{s_{0}}\right). \end{array}$$

In equation (3), *s* denotes the distance from the loud speaker to the left or right ear, *s*_0_ represents the distance selected during sound intensity level calibration, and *D* refers to sound source signal intensity.

The masking effect refers to the phenomenon that the neighbouring sounds with weaker sound intensity levels are masked by strong sounds in the presence of a sound with higher intensity level [16]. Masking model is a method of removing noise interference based on masking effect characteristics [17]. It is assumed that the masking threshold of speech masking noise is *A*(*φ*, *k*), and noise spectrum is expressed by the following equation below.

(4) $$\begin{array}{c} B\left(\varphi ,\text{k}\right)-\overset{\sim }{B}\left(\varphi ,\text{k}\right)\leq A\left(\varphi ,\text{k}\right). \end{array}$$

In equation (4), *B*(*φ*, *k*) represents the noise spectrum and denotes the estimated reduced noise spectrum.

Linear interpolation [18] is used to obtain the calculation method of masking curve model parameter, as shown in the equation below.

(5) $$\begin{array}{c} \left\{\begin{array}{c} y_{u}={\text{k}}_{\text{i}}\left(x+1\right)+c_{i},\\ y_{m}=d_{x}‐10,\\ y_{b}={\text{k}}_{j}\left(x‐1\right)+c_{j}. \end{array}\right. \end{array}$$

In equation (5), *x* refers to the number of the critical band where the frequency is at. *k*_*i*_ and *k*_*j*_ represent the rising slope and falling slope of the simplified masking model function, respectively. *c*_*i*_ and *c*_*j*_ denote the rising intercept and falling intercept of the simplified masking model function, respectively. *d*_*x*_ refers to the sound intensity level of the narrowband signal with critical width with frequency 1 kHz as the center frequency.

The purpose of noise detection is to separate speech segments from background noise segments. A self-adaptive algorithm is a common method of noise detection. However, noise environment does not match actual noise environment in the training process of the algorithm [19]. Hence, it is optimized by the updating of mean and square difference. It is assumed that *X*_1_, *X*_2_, *L*, and *X*_*n*_ are samples of random variables conforming to Gaussian distribution, and then, the estimated Gaussian distribution mean *μ* and square difference *S* of the sample are expressed by the equations below.

(6) $$\begin{array}{c} \mu =\frac{1}{n}\overset{n}{\underset{i=1}{\sum }}X_{n},\\ S=\frac{1}{n}\overset{n}{\underset{i=1}{\sum }}{\left(X_{n}-\mu \right)}^{t}\left(X_{n}-\mu \right). \end{array}$$

After the optimization by the updating of mean and square difference, mean *μ* and square difference *S* are expressed by the equations below.

(7) $$\begin{array}{c} \overset{\sim }{\mu }=\frac{1}{n+1}\left(\overset{n}{\underset{i=1}{\sum }}X_{n}=X\right)=\frac{1}{n+1}\mu +\frac{1}{n+1}X,\\ \begin{array}{c} \overset{\sim }{S}=\frac{1}{n+1}\left[\overset{n}{\underset{i=1}{\sum }}{\left(X_{n}-\mu \right)}^{t}\left(X_{n}-\overset{\sim }{\mu }\right)+{\left(X-\overset{\sim }{\mu }\right)}^{t}\left(X-\overset{\sim }{\mu }\right)\right],\\ =\frac{n}{n+1}S+\frac{n}{{\left(n+1\right)}^{2}}{\left(X-\mu \right)}^{t}\left(X-\mu \right). \end{array} \end{array}$$

In above equations, *X* refers to feature vector, and *n* denotes the number of training samples.

In terms of the initial test tone, the optimal test distance is determined by the test. After that, feature extraction, smoothing, and classification on the test tone are performed. In addition, optimized self-adaptive algorithm is used for noise detection. The test tone is divided into light tone, turbid tone, and noise. The denoising is carried out by an optimized self-adaptive algorithm to analyze if there is a masking effect in the test tone. If there is no masking effect, PTA is performed.  Figure 3 shows the process of speech noise detection below.

### 2.3. Research Objects and Grouping

A total of 46 diabetes patients with SHL diagnosed at the otolaryngology department in Beichen Hospital between August 2019 and November 2021 were selected as the research objects. All of them suffered from unilateral deafness. There were 25 males and 21 females aged between 38 and 77. Their average age was 62.74 ± 3.51. The time range from onset to the first visit was 1 to 15 days with an average of 7.56 ± 1.68 days. All patients previously suffered from diabetes lasting from 0.5 to 22 years. The average disease course was 6.03 ± 2.23 years.

Before and after the treatment, all the patients received conventional ear endoscope, PTA, acoustic immittance, and otoacoustic emission examinations.

Patients were included based on the following standards.

- Patients conforming to the diagnostic standards of *Guidelines for the Diagnosis and Treatment of SHL (2015)* [20]
- Patients previously diagnosed with diabetes and offered drugs to control blood glucose
- Patients with the first onset

Patients were excluded based on the following standards.

- Patients suffering from middle ear lesion, space-occupying lesion, Ménière's disease, and other middle ear and inner ear diseases
- Deaf-mutes, minors, breast feeders, and pregnant and birth-giving women
- Patients with tumours', liver and kidney diseases, and other severe diseases
- Patients with hidden mental diseases or epilepsy
- Patients enrolled in other studies or medications at the same time

All included research objects were randomly divided into the retroauricular group (posterior auricular tympanum injection) and the tympanic group (tympanum injection). Each group included 23 cases. The experimental process had been approved by Beichen Hospital Ethics Committee, and all included research objects had signed informed consent forms.

### 2.4. Different Therapeutic Methods of Diabetes Patients with SHL

All patients were performed on the same vasodilator, neurotrophic, and hyperbaric oxygen drug conventional treatment. Based on these treatments, posterior auricular tympanum injection and tympanum injection of dexamethasone were adopted to treat the patients. Patients in retroauricular group needed to be seated with the affected ear up. After the local disinfection, 1 mL syringe needle was inserted at the upper 1/3 junction of posterior sulcus of the patient's affected ear. 1 mL (5 mg/mL) dexamethasone was injected. After the injection, the affected ear was pressed with a cotton ball for 10 minutes. After that, the affected ear should be kept facing upwards for 30 minutes. The injection needed to be performed 5 times every other day. Patients in tympanic group should be seated with the affected ear up and head tilted back. After the disinfection, tetracaine was used to perform tympanic surface anesthesia. Transperiosteal puncture was performed under ear endoscope with a slender 3 cm needle. Next, 1 mL (5 mg/mL) dexamethasone was injected slowly. After the injection, patients were asked to tilt their heads up 45° and to avoid swallowing and speaking. They needed to hold the position for 30 minutes. The injection should be performed 5 times every other day.

### 2.5. Judgment Methods of Efficacy and Observation Indexes

The literature composed by Herrera et al. (2019) [21] was included as the reference to determining the diagnostic efficacy of SHL. The judgment indexes of the recovery from SHL were as follows. Impaired frequency hearing returned to normal, to healthy ear level, or to the level before the onset. The judgment indexes of significantly effective efficacy were as follows. Impaired frequency hearing was increased by over 30 dB on average. The judgment indexes of effective efficacy were as follows. Impaired frequency hearing was increased by 15 dB to 30 dB on average. The judgment indexes of no efficacy were as follows. Impaired frequency hearing was increased by less than 15 dB on average.

All patients were performed with PTA before and after the treatment. The detection frequency was 250, 500, 1000, 2000, 3000, and 4000 Hz. Besides, the changes in fasting blood glucose (FPG), 2 h postprandial blood glucose (2hPG), and glycosylated hemoglobin (HbA1c) of patients before and after the treatment were monitored for 3 consecutive days. After the treatment course, the differences of tinnitus loudness visual analog scale (VAS) and pain VAS between the patients in two groups were monitored. The statistics on the incidence of adverse drug reactions among the patients in two groups after the treatment was implemented.

### 2.6. Statistical Methods

SPSS22.0 was utilized for data statistics and analysis. Measurement data were expressed by mean ± standard deviation ($\overset{¯}{x}\pm \text{s}$). All quantitative indexes were in accordance with normal distribution with uniform variance. Hence, intergroup variables were compared using independent sample *t* test. Numeration data were denoted by percentage (%) adopting chi-square test. *P* < 0.05 indicated that the differences showed statistical significance.

## 3. Results

This section consists of performance analysis of portable PTA system and comparison of (basic data of included research objects, hear thresholds at different frequencies of patients in two groups, VAS scores between two groups, blood glucose indexes of two groups before and after treatment, clinical efficacy in two groups, and safety of different therapies).

### 3.1. Performance Analysis of a Portable PTA System

The collected speech data of the included research objects were randomly selected. In a soundproof room conforming to national standards, the medical audiometer and the established portable PTA system were used to perform PTA on the patients. Besides, the changes in hear threshold of two audiometry instruments under different frequencies were compared (Figure 4). With different frequencies, the results of hear threshold detected by the medical audiometer and a portable PTA system were generally consistent, and the error was within 2 dB.

The result of monitoring medical audiometer in noise environment was set as the standard to evaluate noise detection performance of self-adaptive algorithm before and after the optimization (Figure 5). With the continuous increase of signal noise ratio (SNR) before and after the optimization, the correct noise detection ratio of the algorithm before and after the optimization both showed an obvious upward trend. With the same SNR, the correct noise detection ratio of the optimized algorithm was obviously higher than that before the optimization.

The changes in hear threshold of medical audiometer and a portable PTA system under noise environment were further compared and analyzed (Figure 6). With different frequencies, the hear thresholds detected by medical audiometer and a portable PTA system after the optimization of the algorithm were generally consistent. However, there was an error around 10 dB between the hear thresholds detected by the algorithm before optimization and medical audiometer.

### 3.2. Comparison of Basic Data of Included Research Objects

Gender proportion, age, height, weight, body mass index (BMI), heart rate (HR), systolic blood pressure (SBP), diastolic blood pressure (DBP), the proportion of patients with left and right deaf ears, diabetes course, and concomitant symptoms of the patients in retroauricular and tympanic groups were compared and analyzed, and the results were displayed in Table 1 below. The comparison of the above indexes showed no statistical differences (*P* > 0.05).

### 3.3. Comparison of Hear Thresholds at Different Frequencies of Patients in Two Groups

The hear thresholds at different frequencies of the patients in retroauricular and tympanic groups before and after the treatment were compared and analyzed (Figure 7). No statistical differences were found in the comparison of the hear thresholds at different frequencies of the patients in the two groups before and after the treatment (*P* > 0.05). After the adoption of different therapeutic methods, the hear thresholds at different frequencies in the two groups were both reduced compared with those before the treatment (*P* < 0.05). The comparison of the hear thresholds at different frequencies in the two groups after the treatment showed no statistical differences (*P* > 0.05).

The average PTA of the patients in the retroauricular and the tympanic groups before and after treatment was compared and analyzed (Figure 8). The comparison of the average PTA of the patients in two groups before treatment showed no statistical differences (*P* > 0.05). After the adoption of different therapeutic methods, the average PTA in the two groups was both decreased and compared with those before treatment (*P* < 0.05). No statistical differences were spotted by the comparison of the average PTA in the two groups after treatment (*P* > 0.05).

### 3.4. Comparison of VAS Scores between Two Groups

The decreased tinnitus VAS values and pain VAS scores of the patients in retroauricular and tympanic groups after treatment were compared and analyzed (Figure 9). After treatment, the decreased tinnitus VAS values of retroauricular and tympanic groups were 4.63 ± 0.56 and 2.27 ± 0.33, respectively. The decreased tinnitus VAS values of the former group was significantly higher than that of the latter one (*P* < 0.01). The pain VAS scores in retroauricular and tympanic groups were 2.95 ± 0.38 and 6.02 ± 0.64, respectively. The pain VAS scores of the former group was remarkably lower than that of the latter group. The comparison between two groups showed extremely notable differences (*P* < 0.001).

### 3.5. Comparison of Blood Glucose Indexes of Two Groups before and after Treatment

FPG, 2hPG, and HbA1c of the patients in retroauricular and tympanic groups before and after treatment were compared and analyzed (Figure 10). No statistical difference was found by the comparison of FPG and 2hPG in the two groups before and after treatment (*P* > 0.05). After treatment, HbA1c in the two groups was both increased compared with those before treatment. However, the difference demonstrated no statistical significance (*P* > 0.05). The comparison of HbA1c in the two groups before and after treatment had no statistical differences (*P* > 0.05).

### 3.6. Comparison of Clinical Efficacy in Two Groups

The statistics and analysis of the proportions of cured, significantly effective, effective, and ineffective patients and the total effective rate in retroauricular and tympanic groups were carried out (Figure 11). The number of cured, significantly effective, effective, ineffective patients, and the total effective rate in retroauricular group were 6 (26.09%), 7 (30.43%), 8 (34.78%), 2 (8.70%), and 21 (91.30%), respectively. Those in tympanic group were 7 (30.43%), 6 (26.09%), 9 (39.13%), 1 (4.35%), and 22 (95.65%), respectively. The comparison of the proportions of cured, significantly effective, effective, and ineffective patients. The total effective rate in retroauricular and tympanic groups after treatment showed no statistical differences (*P* > 0.05).

### 3.7. Comparison of Safety of Different Therapies

The statistics and analysis of the adverse reactions among the patients in retroauricular and tympanic groups after treatment were carried out (Figure 12). In retroauricular group, 1 patient suffered from vertigo and 1 suffered from otalgia after treatment (4.35%). In tympanic group, there were 3 cases infected (13.04%), 2 with vertigo (8.70%), 1 suffering from periosteal perforation, 1 with otalgia, 1 with ear numbness, and 1 suffering from periosteal errhysis (4.35%). The incidence of adverse reactions in retroauricular and tympanic groups after treatment amounted to 8.70% (2 cases) and 39.13% (9 cases), respectively. The incidence of adverse reaction after treatment of the latter group was dramatically higher than that of the former one. The comparison between two groups indicated extremely remarkable differences (*P* < 0.001).

## 4. Discussion

Portable PTA system shows noise masking effect. The audiometry results cannot get the accurate hear threshold of otological normal people [22]. A masking model and an optimized self-adaptive algorithm were adopted to detect and reduce noise, which showed that the hear threshold results of medical audiometer and portable PTA system at different frequencies were generally consistent, and the error was within 2 dB. Under the same SNR, the correct noise detection rate of the optimized algorithm was evidently higher than that of the algorithm before optimization. However, there was an error of around 10 dB between the hear thresholds detected by the algorithm before optimization and medical audiometer. The above results revealed that the presence of noise increased the hear threshold of the subjects, which was consistent with PTA results in hospital soundproof room [23]. It was demonstrated that portable PTA system showed good detection reliability both in mute and noise conditions with accurate audiometry results.

At present, the cause of SHL is unknown. The incidence of SHL among diabetes patients with SHL may be correlated with the capillary vessel lesion of diabetes patients' inner ears [24], the increase in microcirculation viscosity of inner ears [25], and the metabolic disorder of inner ears [26]. Multiple mechanisms disrupt the balance of body blood coagulation, anticoagulation, and fibrinolysis [27]. Consequently, the hearing impairment among the patients becomes severe, and SHL is induced. Glucocorticoid shows anti-inflammation, vasospasm relief, local edema alleviation, and other effects. It can remarkably improve inner ear circulation microenvironment and is the first choice for SHL treatment [28]. Administration methods include systemic administration and local administration. The systemic administration method for diabetes patients with SHL causes the increase of blood glucose concentration, the aggravation of diabetes, and even some serious complications, such as diabetic ketoacidosis [29]. Hence, local administration method is the first choice for treating diabetes patients with SHL. Some researchers treat diabetes patients with SH by systemic, inner tympanum, and posterior auricular administration methods. The results showed that the three therapies demonstrated good efficacy, and no statistical differences existed among the effective rate of the treatment [30]. Posterior auricular and tympanum injection of dexamethasone were utilized to treat diabetes patients with SHL. The results indicated that the hear thresholds and average PTA of the patients in retroauricular and tympanic groups at different frequencies were both decreased compared with those before treatment (*P* < 0.05). After treatment, no statistical differences were shown by the comparison of the hear thresholds, the proportions of cured, significantly effective, effective, ineffective patients, and the total effective rate among the patients in retroauricular and tympanic groups at different frequencies (*P* > 0.05). The result demonstrated that the comparison of the total effective rate and efficacy of the treatment of diabetes patients with SHL by posterior auricular and tympanum injection of dexamethasone showed no statistical differences. The outcome was consistent with the research result obtained by Jia et al. (2019) [8]. The further analysis of pain and the incidence of adverse reactions among patients after the treatment by the two methods revealed that the VAS value in the retroauricular group decreased more remarkably than that in the tympanic group (*P* < 0.01), and pain VAS score was obviously lower than that in tympanic group (*P* < 0.001). The results indicated that tinnitus VAS score and pain VAS score among the patients in retroauricular group could be significantly reduced, which might be caused by the utilization of lidocaine during the injection. The local anesthesia could alleviate patients' pain. Besides, it was pointed out in some studies that tympanum administration method enabled the drug to enter the inner ears through fenestra cochleae, which resulted in the difficulties in controlling dosage, duration, and absorption effect and the significant differences among individuals [31]. The results demonstrated that the incidence of adverse reactions in tympanic group after treatment was obviously higher than that in retroauricular group (*P* < 0.001), which indicated that inner ear administration method could remarkably reduce the incidence of adverse reactions. The outcome was similar to the research result obtained by Zhou et al. (2017) [32]. To conclude, posterior auricular and tympanum injection of dexamethasone could both effectively improve the strength of diabetes patients with SHL with little influence on blood glucose concentration. In contrast to tympanum injection, posterior auricular injection caused fewer adverse reactions and pains. Hence, it showed the potential values in clinical popularization and application.

## 5. Conclusions

Based on mobile terminals, portable PTA system was established preliminarily, and its noise processing method was discussed. Besides, the efficacy of tympanum injection and posterior auricular injection in SHL with diabetes was compared, and the audiometry result of portable PTA system was accurate. Posterior auricular injection caused fewer adverse reactions and pains. However, there are still some disadvantages in the research. The included sample size was limited, and it needed to be enlarged at the later stage. In addition, rigorous randomized controlled studies should be adopted to further validate the efficacy of different therapies. In brief, portable PTA system and its noise processing method were established. Posterior auricular injection showed the potential application values in the treatment of SHL with diabetes, which provided a new idea and reference basis for the diagnosis and treatment of SHL patients with diabetes.

## Figures and Tables

**Figure 1:** Overall framework of a mobile terminal-based portable PTA system.

**Figure 2:** Application process of a portable PTA system.

**Figure 3:** Process of speech noise detection.

**Figure 4:** Comparison of PTA results of different audiometry systems.

**Figure 5:** Comparison of noise detection performance of self-adaptive algorithm before and after optimization.

**Figure 6:** Comparison of audiometry results of different audiometry systems in different noise conditions.

**Figure 7:** Comparison of hear thresholds at different frequencies in two groups. (∗ indicated that the comparison with those before treatment showed statistical differences, *P* < 0.05)

**Figure 8:** Comparison of the average PTA in the two groups. (∗ indicated that the comparison with those before treatment showed statistical differences, *P* < 0.05).

**Figure 9:** Comparison of VAS scores between two groups. (∗∗ indicated that the comparison with retroauricular group showed significant differences, *P* < 0.01. ∗∗∗ revealed that the comparison with retroauricular demonstrated extremely remarkable differences, *P* < 0.001)

**Figure 10:** Comparison of blood glucose indexes in two groups before and after treatment.

**Figure 11:** Comparison of clinical efficacy between two groups.

**Figure 12:** Comparison of incidence of adverse reactions of different therapies. (∗ showed the comparison with retroauricular group indicated statistical differences, *P* < 0.05. ∗∗ revealed that the comparison with retroauricular group demonstrated significant differences, *P* < 0.01. ∗∗∗ indicated that the comparison with retroauricular group showed extremely notable differences, *P* < 0.001).

**Table 1:** Comparison of basic data of included research objects.

Factors	Retroauricular group (*n* = 23)	Tympanic group (*n* = 23)	*χ* ^2^/*t* value	*P* value
Gender (case (%))			0.554	0.648
Male	13 (56.52%)	12 (52.17%)		
Female	10 (43.48%)	11 (47.83%)		
Age (years old)	63.03 ± 5.35	62.58 ± 6.21	1.445	0.727
Weight (kg)	61.18 ± 7.08	61.39 ± 10.02	1.127	0.924
Height (cm)	166.83 ± 12.16	165.28 ± 12.94	1.156	0.916
BMI (kg/m^2)^	22.23 ± 3.02	22.07 ± 2.87	1.525	0.653
HR (beat/min)	64.06 ± 7.03	63.83 ± 6.85	1.285	0.687
SBP (mmHg)	122.96 ± 11.87	123.18 ± 12.44	1.042	0.813
DBP (mmHg)	81.85 ± 9.16	81.44 ± 8.97	1.134	0.809
Deaf ears (case (%))			0.611	0.627
Left	12 (52.17%)	13 (56.52%)		
Right	11 (47.83%)	10 (43.48%)		
Diabetes course (year)	5.88 ± 1.05	6.06 ± 0.98	1.153	0.815
Concomitant symptoms (case (%))			0.201	0.928
Vertigo	8 (34.78%)	9 (39.13%)		
Tinnitus	18 (78.26%)	15 (65.22%)		
Ear stuffy feeling	14 (60.87%)	12 (52.17%)		

## Data Availability

The experimental data used to support the findings of this study are available from the corresponding author upon request.
